The article "Blockage of Fibronectin 1 Ameliorates Myocardial Ischemia/Reperfusion Injury in Association with Activation of AMP-LKB1-AMPK Signaling Pathway" was published in 2022. Journal: Oxid Med Cell Longev.

# Blockage of Fibronectin 1 Ameliorates Myocardial Ischemia/Reperfusion Injury in Association with Activation of AMP-LKB1-AMPK Signaling Pathway

**DOI:** 10.1155/2022/6196173

**Published:** 2022-05-12

**Authors:** Yun-Long Zhang, Pang-Bo Li, Xiao Han, Bo Zhang, Hui-Hua Li

**Affiliations:** ^1^Department of Emergency Medicine, Beijing Key Laboratory of Cardiopulmonary Cerebral Resuscitation, Beijing Chao-Yang Hospital, Capital Medical University, Beijing 100020, China; ^2^Department of Cardiology, Institute of Cardiovascular Diseases, First Affiliated Hospital of Dalian Medical University, Dalian 116011, China

## Abstract

Myocardial ischemia/reperfusion injury (I/RI) is closely associated with energy substrate metabolism. Fibronectin 1 (Fn1) was markedly elevated in the heart of I/R pigs and ischemic patients, but its role in myocardial I/RI is controversial and the precise mechanism involved remains elusive. Herein, we tested whether blockage of Fn1 with its inhibitor (fibronectin tetrapeptide, RGDS) would alleviate myocardial I/RI. Wild-type (WT) mice were administered with RGDS once 3 h before I/R operation and once at 24 or 48 h postreperfusion, and sacrificed at 24 or 72 h post-I/R, respectively. Cardiac function was evaluated by echocardiography. Myocardial infarction size, apoptosis, fibrosis, and inflammation were examined via histological staining. Uptake of glucose and fatty acids were detected by positron emission tomography (PET) and computer tomography (CT) with [^18^F]-2-fluoro-2-deoxy-D-glucose (FDG) and [^18^F]-fluoro-6-thia-heptadecanoic acid (FTHA), respectively. Our results showed that administration of RGDS to mice remarkably limited the I/R-induced myocardial infarct size, myocyte apoptosis, inflammation, oxidative stress, and fibrosis and improved cardiac contractile dysfunction. These protective effects were associated with upregulation of the AMP/ATP ratio and the activation of LKB1-AMPK signaling, which subsequently increased AS160-GLUT4-mediated glucose and fatty acid uptake, improved mitochondrial dynamic imbalance, and inactivated TGF-*β* and NF-*κ*B signals in the I/R heart. In conclusion, the current study identified that blocking Fn1 protects against myocardial I/RI likely through activating the LKB1-AMPK-dependent signals and highlights that inhibition of Fn1 may be a novel therapeutic option for treating ischemic heart diseases.

## 1. Introduction

Coronary artery disease (CAD) frequently leads to heart failure (HF), a leading cause of death worldwide. The major pathological manifestation of CAD is cardiac myocyte death due to ischemia/reperfusion injury (I/RI). Thus, swiftly restoring blood flow to ischemic tissues can reestablish energy production and cell survival and limit myocardial damage. Paradoxically, sudden reperfusion also causes myocyte death and cardiac arrest [1, 2]. Therefore, it is imperative to discover new therapy targets to protect against I/R-induced myocardial injury and dysfunction in patients with CAD.

Accumulating evidence has revealed that potential mediators of myocardial I/RI mainly include cell death (such as necrosis, apoptosis, and autophagy), oxidative stress, and inflammation [3–5]. In recent years, mitochondrial dysfunction, particularly impairment in energy and substrate utilization, such as glucose and fatty acid (FA) has been reported as a key determinant of apoptosis, a major form of cell death in myocardial I/RI [4]. Moreover, alteration of mitochondrial dynamics, impairment of electron transport chain complex activity, calcium overload, and increased reactive oxygen species (ROS) production also significantly contribute to I/R-induced mitochondrial dysfunction [4]. Importantly, 5′AMP-activated protein kinase (AMPK) plays a key role in regulating glucose and FA metabolism, mitochondrial function, and cellular apoptosis in the ischemic myocardium [6, 7]. Interestingly, some interventions against these signals have been demonstrated to prevent or improve myocardial I/RI in animal models, but none have been clinically validated as an effective treatment in patients [8–10].

Fn1 is a glycoprotein involved in cellular adhesion, growth, and angiogenesis [11]. Fn1 is produced by various cell types, including endothelial cells, cardiomyocytes, and myofibroblasts [12]. Previous results have indicated that Fn1 expression is upregulated in the I/R heart tissues of pigs and in patients with ischemic or dilated cardiomyopathy. Interestingly, Fn1 polymerization is required for collagen deposition and plays a critical role in I/R-induced myocardial fibrosis, inflammation, and vasculogenesis after infarction [13–16]. However, its role is controversial, and the molecular mechanism involved in myocardial I/R remains to be explored.

In this study, using Fn1 inhibitor (fibronectin tetrapeptide, RGDS), we focused on investigating the role of Fn1 in I/R-triggered cardiac myocyte apoptosis and impairment of energy metabolism and elucidated the potential mechanism in mice. We demonstrated that Fn1 expression was significantly upregulated in the I/R heart. Administration of mice with RGDS markedly ameliorated I/R-induced cardiac infarction, myocyte apoptosis, inflammation, oxidative stress, and fibrosis likely via by activating the AMP-LKB1-AMPK-dependent signaling pathways.

## 2. Material and Methods

### 2.1. Ischemia/Reperfusion Model and Treatment

Wild-type (WT, male, and C57BL/6J) mice at age of 10 weeks old (weighing 20–23 g) were obtained from SPF Biotechnology Co., Ltd. (Beijing). The mice were kept in a conditioned room (24-25°C) and 12-h light/dark and were allowed free access to the diets and water. An I/R murine model was established by ligating the left anterior descending coronary artery (LAD) as described [17]. Briefly, mice were anesthetized with pentobarbital sodium (60 mg/kg body weight (BW)). A 6-0 silk suture slipknot was placed around the LAD coronary artery for 30 min (ischemia) and then released the slipknot to allow reperfusion for 24-72 hours. Control mice underwent a sham operation without LDA ligation. Meanwhile, buprenorphine hydrochloride (0.01 mg/kg, Sigma-Aldrich) was administered as an intraoperative analgesic.

To understand the expression pattern of Fn1 during myocardial I/RI, animals were randomly divided into 4 groups, Sham, I/R6h, I/R24h, and I/R72h (*n* = 4 mice per group). To test the effect of Fn1 inhibitor (RGDS peptide; H-Arg-Gly-Asp-Ser-OH) on myocardial I/RI, animals were randomly divided into 6 groups, sham (saline, RGDS), I/R24h (saline, RGDS), and I/R72h (saline, RGDS) (*n* = 42 mice per group). RGDS and Arg-Gly-Glu-Ser (RGES, a scramble control) were from Sigma-Aldrich (St. Louis, MO). Mice in the sham+RGDS and I/R + RGDS groups were injected intraperitoneally with RGDS in saline (5 mg/kg BW) as previously described [18, 19]. RGDS were administered once 3 h before I/R operation and once at 24 or 48 h postreperfusion and sacrificed at 24 or 72 h post-I/R. An equal amount of RGES (5 mg/kg) in saline (hereafter referred to as: saline) was administered to the sham+saline and I/R + saline groups as controls. All mice were deeply euthanized with 2.5% 2,2,2-tribromoethanol and hearts were prepared for further experiments. This study and experimental procedures were approved and performed in accordance with the Animal Care and Use Committee of Capital Medical University (AEEI-2020-155) and conformed to the Guide for the Care and Use of Laboratory Animals (the U.S. National Institutes of Health).

### 2.2. Echocardiography

Animals (*n* = 8 per group) were anesthetized with isoflurane at a dose of 1.5-2.0%. Cardiac function was evaluated with echocardiography using a Vevo 1100 high-resolution imaging system (Visual Sonics Inc.) The parameters for left ventricular internal dimension at end-diastole (LVIDd) or at end-systole (LVIDs) as well as the percentage of ejection fraction (EF%) or fractional shortening (FS%) were calculated for all mice as described previously [17].

### 2.3. PET/CT Imaging

Glucose and FA metabolism in the heart of mice (*n* = 3 per group) were evaluated by positron emission tomography (PET) with [^18^F]-2-fluoro-2-deoxy-D-glucose (FDG) and [^18^F]-fluoro-6-thia-heptadecanoic acid (FTHA), which reflect glucose uptake and *β*-oxidation rate of free FAs in the heart, respectively [20–22]. Scans were acquired with a Super Nova SNPC-103 Micro PET/CT scanner (Pingseng Healthcare Inc.). Static PET/CT images were obtained 40 min after the injection of [^18^F]-FDG (180-220 MBq; 24 or 72 h after reperfusion) and [^18^F]-FTHA (a free FA for myocardial PET imaging, 180-250 MBq; 24 or 72 h after reperfusion), with an acquisition time of 40 min. Images were reconstructed using the Pingseng Avatar software (version 1.4.0). Next, the acquired data were Fourier-rebinned in six time frames (2 × 300 s, 2 × 600 s, 2 × 1800 s) and reconstructed using a three-dimensional ordered-subsets expectation maximum algorithm (3D-OSEM). For the quantification of tracer uptake, two-dimensional (2D) circular regions of interest were placed on coronal PET/CT images of the hearts, and the standard uptake values (SUVs) were recorded.

### 2.4. Measurement of Infarct Area

At the end of the experiment, mice (*n* = 5/group) were injected intraperitoneally with an overdose of pentobarbital sodium (100 mg/kg) and then flushed transcardially with saline solution. The nonischemic or infarct region of the heart was detected as described previously [17]. Briefly, after anesthesia, the LAD was ligated, and 200 *μ*l of 1% Evans blue dye (Sigma-Aldrich) was infused into the left ventricle from the apex cordis. The heart was removed and quickly frozen at −20°C for 15 min and then cut into 4 equal pieces (~2 mm) from apex to base. Each slice was weighed and incubated in 1% 2,3,5-triphenyltetrazolium chloride (TTC) solution at 37°C for 20 min. These slices were fixed in 4% paraformaldehyde for 24 h and then analyzed using the Image-ProPlus software. Three main zones in the stained heart sections are distinguishable: white: infarct tissue; red: at-risk tissue; blue: nonrisk tissue. The percentage of total ischemic areas = (infarct + at − risk) areas/total myocardial areas; the percentage of necrotic areas = infarct areas/(infarct + at − risk) areas.

### 2.5. Histological Analysis

Cardiac tissues (*n* = 5-6 per group) were fixed in 10% formalin solution overnight and then embedded in paraffin. A 5 *μ*m thick section of tissue was cut serially and stained with anti-Mac-2 antibody or Masson's trichrome, respectively [17, 23]. To detect cardiomyocyte apoptosis, sections (*n* = 5 per group) were stained with a TUNEL Apoptosis Detection (red) Kit (Roche, IN, USA) as per the manufacturer's protocols. 10-12 visual fields were randomly selected from each heart sample. The number of TUNEL-positive cells visualized in fluorescein green (*α*-actinin) to the number of DAPI-stained nuclei was determined and represented the percentages of apoptotic cells per group [17]. For reactive oxygen species (ROS) analysis, heart cryosections (5 *μ*m thick) were stained with 1 *μ*mol/l dihydroethidine (DHE) in PBS buffer at 37°C for 30 minutes. The images were obtained from over 10 random fields for each sample using a Labophot 2 microscope (Nikon, Tokyo). The levels of 8-hydroxy-2′-deoxyguanosine (8-OHdG) in myocardial tissue were detected by ELISA kit (CCA660Ge, Cloud-Clone Corporation, TX).

### 2.6. Quantitative Real-Time PCR Analysis

Total RNA from the border zone of the I/R-treated heart (*n* = 4 per group) was extracted with the TRIzol (Invitrogen) following the manufacturer's protocols. Equal amount (1 *μ*g) of total RNA was used to synthesize the cDNA using the RT Enzyme mix (Accurate Biotechnology Co., Ltd.). The mRNA levels of Fn1 were measured with quantitative real-time PCR (qPCR) using a PCR thermocycler (Bio-Rad). The value was normalized to that of GAPDH. The primers for Fn1: 3′-ATCCAGTCCACAGCCATTCC-5′ (forward) and 3′-GGAAGGGTAACCAGTTGGGG-5′ (reverse). GAPDH: 3′-GGTTGTCTCCTGCGACTTCA-5′ (forward) and 3′-GGTGGTCCAGGGTTTCTTACTC-5′ (reverse). Collagen I: 3′-GAGTACTGGATCGACCCTAACCA-5′ (forward) and 3′-GACGGCTGAGTAGGGAACACA-5′ (reverse) and Collagen III: 3′-TCCCCTGGAATCTGTGAATC-5′ (forward) and 3′-TGAGTCGAATTGGGGAGAAT-5′ (reverse).

### 2.7. Western Blot Analysis

Proteins were isolated from the border zone of the I/R cardiac tissues (*n* = 4 per group) with RIPA lysis buffer containing the protease inhibitor cocktail. The protein level was determined with a BCA protein assay kit according to the manufacturer's protocols. Equal amount (50 *μ*g) of proteins was subjected to 10% sodium dodecylsulfate-polyacrylamide- (SDS-) polyacrylamide gel electrophoresis (PAGE) gel and then transferred to a polyvinylidene fluoride (PVDF) membrane (Millipore). The latter were immunoblotted with primary antibodies (Table 1) at 4°C overnight. All blots' densitometric analyses were performed with the Image J Software (NIH) and normalized to GAPDH expression level as described [17].

### 2.8. Measurement of ATP and AMP Content

ATP and AMP levels were measured using an ATP or AMP Assay Kit (ab83355, ab273275; Abcam, Cambridge, MA), respectively, according to the manufacturer's protocols. In short, cardiac tissues (10 mg, *n* = 5 per group) were washed with cold PBS then resuspended in 100 *μ*l of ATP or AMP assay buffer, and subsequently centrifuged at 13,000 x g (4°C). The supernatants were then incubated with the ATP probe for 30 minutes at room temperature or the reaction mix for 60 minutes at 37°C. The absorbance of sample at 570 nm was detected with an automatic microplate reader (Infinite, M1000 PRO, Tecan Inc.).

### 2.9. Study Patients

We explored all-comers of patients with ST-segment elevation myocardial infarction (STEMI) treated with percutaneous coronary intervention (PCI) and age- and sex-matched control subjects in a monocentric clinical cohort between November 2021 and December 2021. STEMI patients were diagnosed according to the 2020 ESC Guidelines [24]. The blood samples were collected from 30 patients with STEMI treated with PCI and 30 control subjects. Plasma Fn1 protein level was measured by ELISA assay kit (E-EL-H0179c, Elabscience) according to the manufacturer's instructions. The study was approved by the First Hospital Ethics Committee of Dalian Medical University (No. PJ-KS-KY-2021-156) and conformed with the principles outline in the Declaration of Helsinki. Written informed consent was obtained from each patient.

### 2.10. Statistical Analysis

All results were expressed as mean ± SEM. Statistical analyses were conducted with GraphPad Prism 7. Groups were compared using the two-sample Student's *t* test or the nonparametric Mann–Whitney *U* test. Multivariable logistic regression models were used to evaluate the association of human STEMI and plasma Fn1 level while adjusting for age, systolic blood pressure, HDL cholesterol, creatinemia, blood glucose, platelet, and uric acid. A *P* value < 0.05 was considered statistically significant.

## 3. Results

### 3.1. Fn1 Was Upregulated in I/R Mouse Heart and Patients

To understand the expression pattern of Fn1 during myocardial I/RI, we first performed a qPCR analysis of the cardiac tissues at 6, 24, and 72 hours after I/R operation. Our results revealed that Fn1 mRNA expression was time-dependently (6-72 h) upregulated by 2.2- to 16.6-fold in the I/R heart group compared with the sham control (Figure 1(a)). The increased Fn1 protein levels at different time points (1.1- to 2.7-fold) were confirmed in the I/R hearts by immunoblotting analyses (Figure 1(b)).

To examine whether Fn1 is associated with human myocardial I/R injury, we examined Fn1 level in the blood and found that plasma Fn1 level was significantly increased 2-fold in STEMI patients treated with PCI compared with controls (Figure 1(c)). The baseline characteristics and cardiac risk factors of healthy control subjects and STEMI patients are shown in Table 2. We then analyzed the relation of serum Fn1 level in patients with STEMI by simple crosstabulation and the calculations of odds ratios (ORs). After adjustment for sex, age, and cardiovascular risk factors, a significant relationship was found between Fn1 level (OR, 23.683) and STEMI (*P* = 0.032; Table 3). Overall, these results suggest that increased Fn1 may contribute to the pathogenesis of myocardial I/RI.

### 3.2. Blockage of Fn1 Ameliorated I/R-Induced Myocardial Dysfunction

To explore the functional role of Fn1 in the regulation of myocardial I/RI, we administered Fn1 inhibitor (RGDS peptide) to WT mice daily and then subjected them to I/R for 24 and 72 h (Figures 2(a) and 2(b)). Echocardiography displayed that the I/R-operated mice had a time-dependent reduction in cardiac contractile function, as reflected by decreased left ventricular ejection fraction (EF, 33% and 25% for 24 and 72 h, respectively) and fractional shortening (FS, 16% and 12% for 24 and 72 h, respectively), compared with sham-operated controls. However, blockage of Fn1 by RGDS markedly reversed this effect (EF, 45% and 36%; FS, 22% and 18%) (Figures 2(c) and 2(d)). Besides, I/R-induced increase of cardiac chamber dimensions, as indicated by LVIDs, systolic left ventricular internal diameters (LVIDs), and diastolic left ventricular internal diameters (LVIDd), was considerably reduced in RGDS-treated mice (Figure 2(d)).

### 3.3. Blockage of Fn1 Reduced I/R-Induced Cardiac Infarct Size and Myocyte Apoptosis

Since cardiomyocytes are the main cells of related to cardiac function, their loss worsens cardiac contractile function. Therefore, we performed TTC and Evan's Blue staining as well as TUNEL assay, which revealed that there was similar areas at risk (AARs) among groups, but the infarct area/AAR ratio (29% and 52%) and the percentage of TUNEL-positive cardiac myocytes (1.2% and 2.3%) in saline-treated controls were markedly lower in RGDS-administered mice (infarct area/AAR ratio, 9% and 23%; apoptosis, 0.42% and 0.51%) at 24 and 72 h of reperfusion, respectively (Figures 3(a) and 3(b)). Immunoblotting established that the I/R-mediated increase of Bax/Bcl-2 ratio and cleaved caspase-3 protein in saline-treated hearts were also substantially attenuated in RGDS-treated hearts at different reperfusion time points (Figure 3(c)).

### 3.4. Blockage of Fn1 Suppresses I/R-Induced Cardiac Inflammation and Fibrosis

Inflammation is a hallmark of cardiac injury after I/R. We then performed immunohistochemical staining that indicated that the I/R stress caused a significant increase of infiltration of Mac-2-positive macrophages in the saline-treated hearts (10% and 19%) compared with sham control (3.7%), which was remarkably reduced in RGDS-treated hearts (6.4% and 10.3%) at 24 and 72 h of reperfusion (Figure 4(a)). Oxidative stress plays a critical role in cardiac I/RI. DHE staining revealed that the I/R operation resulted in a marked upregulation of ROS production in the saline-treated hearts (7.4- and 17.8-fold) compared sham-treated hearts, but this increase was time-dependently reduced to 2.9- and 6.5-fold in RGDS-treat hearts at 24 and 72 h of reperfusion, respectively (Figure 4(b)). Moreover, I/R for 24 and 72 h significantly upregulated 8-OHdG level (a marker of mitochondrial DNA oxidative damage) in the heart tissue (1.3- and 1.6-fold) compared with sham hearts, whereas this increase was markedly reduced by 21% and 25% in RGDS treated mice (Figure 4(d)). Furthermore, Masson trichrome staining showed that I/R-induced increase of myocardial fibrotic area (14.3% and 40.1% for 24 and 72 h, respectively) in the saline-treated hearts was dramatically reduced in RGDS-treated hearts by 6- and 13.1-fold, respectively (Figure 4(c)). Accordingly, I/R-induced upregulation of collagen I and collagen III (well-characterized markers of fibrosis) mRNA levels in the saline-treated hearts was lower than in RGDS-treated hearts after 24 and 72 h of reperfusion, respectively (Figure 4(e)). In addition, the protein levels of TGF-*β*1 (a critical regulator of tissue fibrosis) and NF-*κ*B-p65 (a key transcription factor for inflammatory cytokine expression) in saline-treated mice were greatly lower in RGDS-treated hearts at different time points after reperfusion (Figure 4(f)).

### 3.5. Inhibition of Fn1 Restored Glucose and Fatty Acid Uptake

Glucose and FA metabolism alteration is closely associated with myocyte apoptosis and cardiac dysfunction after I/R [6, 25]. To examine whether Fn1 affects energy metabolism in the I/R myocardium, we measured cardiac glucose and FA uptakes at 24 or 72 h after reperfusion using PET with [^18^F]-FDG or [^18^F]-FTHA (reflecting the betaoxidation rate of free FAs, respectively [21, 22]. As illustrated in Figures 5(a) and 5(b), I/R time-dependently decreased myocardial glucose (56% and 42% for 24 and 72 h, respectively) and FA uptake (43% and 34% for 24 and 72 h, respectively), as reflected by decreased left ventricular (LV)/blood SUVs, in saline-treated mice compared with sham and saline-treated controls. Conversely, this effect was largely restored in RGDS-treated hearts (glucose: 78% and 58%; FA: 70% and 60%).

### 3.6. Inhibition of Fn1 Activated AMP/ATP -LKB1-AMPK Pathway

Since AMPK signaling plays a key role in protection of myocardial I/RI, we next examined the activation of LKB1-AMPK signaling in saline or RGDS- and I/R-cotreated hearts. Immunoblotting revealed that I/R resulted in a marked downregulation of p-LKB1 (Ser428) and p-AMPK (T172) protein levels in saline-treated mice, but this decrease was significantly restored in RGDS-treated hearts (Figures 6(a) and 6(b)). Accordingly, I/R-mediated decrease of GLUT4 (a critical regulator of glucose uptake), AS160 (a regulator of GLUT-4 intramyocellular redistribution) and Mfn1/2 (critical regulators of mitochondrial fusion) and upregulation of p-Drp1(S616) and total Drp1 (a key regulator for mitochondrial fission) in saline-treated mice were also remarkably reversed in RGDS-treated hearts (Figures 6(a) and 6(b)). In addition, the AMP/ATP ratio (a critical regulator for the activation of LKB1-AMPK signaling) in RGDS-treated hearts was markedly higher than in saline-treated mice (Figure 6(c)). Thus, blocking Fn1 ameliorates myocardial I/RI in associated with activation of AMP/ATP-LKB1-AMPK signaling and increase of glucose and FA uptake as well as improvement of mitochondrial dynamics.

## 4. Discussion

Here, our results demonstrate for the first time that I/R significantly upregulated Fn1 expression and production in mouse hearts and patients with STEMI. Conversely, administration of Fn1 inhibitor RGDS to mice remarkably ameliorated I/R-induced myocardial infarct size, myocyte apoptosis, inflammation, oxidative stress, and fibrosis, which were associated with inhibition of AMP/ATP-LKB1-AMPK-dependent mechanisms (Figure 7). Thus, these findings indicate that blocking Fn1 may be new therapeutic target for treating myocardial I/RI.

Fn1 is a high-molecular-weight glycoprotein present in plasma as a soluble dimer and as a dimer or multimer at the cell surface and extracellular matrix [11]. Upregulation of Fn1 expression has been consistently observed in diverse cardiovascular tissues under pathological conditions. For example, Fn1 expression is markedly increased in the aorta, atria, and ventricles of deoxycorticosterone-salt or L-triiodothyronine-treated rats and spontaneously hypertensive rats [26, 27]. Interestingly, the Fn1 level was also highly upregulated in the infarct tissue compared with the remote and noninfarcted tissues in pigs after I/R [13]. Consequently, we confirmed that Fn1 was time-dependently increased in the I/R hearts of mice (Figures 1(a) and 1(b)) and further identified that serum Fn1 in STEMI patients was significantly higher than in normal controls (Figure 1(c)), suggesting that increased Fn1 may be involved in the regulation of I/RI. However, the effect of Fn1 on myocardial infarction and I/RI remains controversial. For example, inhibition of Fn1 polymerization or ablation of Fn1 in cardiac fibroblasts attenuates cardiac fibrosis, inflammation, and cardiac dysfunction after I/RI [15]. Conversely, genetic ablation of Fn1 blunts the proliferation and survival of cardiac progenitor cells and attenuates vasculogenesis and cardiogenesis, leading to a continuous decline in cardiac function during recovery after 12 weeks of myocardial infarction [14]. Thus, it is imperative to clearly verify the role of Fn1 in the regulation of myocardial I/RI and elucidate the underlying mechanisms. In this study, using Fn1 inhibitor in an I/R mouse model, we demonstrated that blockage of Fn1 in mice significantly reduced myocardial infarction, cardiomyocyte apoptosis, inflammation, oxidative stress, and fibrosis, leading to improved contractile dysfunction after I/RI (Figures 2–4), supporting the findings that inhibition of Fn1 improves myocardial I/RI.

Myocardial I/RI is frequently accompanied by profound changes in mitochondrial dysfunction and energy substrate (glucose and FA) metabolism. Notably, AMPK is a key energy sensor that critically regulates uptake of glucose, glycolysis, and FA oxidation during I/RI in diverse tissues [7, 25]. Increasing evidence demonstrates that AMPK activation displays beneficial effects against I/RI in the heart and other organs via multiple mechanisms, including increasing energy metabolism, reducing oxidative stress, and improving mitochondrial dysfunction and inflammatory response [7, 25]. Along these lines, the modulation of AMPK activation may represent a promising cardioprotective option for the treatment of this disease. To determine whether Fn1 promoted myocardial I/RI by regulating LKB1-AMPK-mediated energy metabolism, we examined the AMP/ATP level and measured the glucose and FA uptake using PET with [^18^F]-FDG and FTHA, respectively, and observed that inhibition of Fn1 significantly restored the I/R-induced decrease in the uptake of glucose and FAs (Figure 5), accompanied by increased AMP/ATP ratio, activation of LKB1-AMPK, and the upregulation of GLUT4 and AS160 proteins (Figure 6). These findings imply that inhibition of Fn1 can enhance LKB1-AMPK signaling-mediated energy metabolism, which ameliorates I/R-induced cardiac myocyte apoptosis and dysfunction.

Accumulating evidence demonstrates that AMPK also exerts a key role in maintaining mitochondrial dynamics, redox homeostasis, inflammation, and fibrosis through regulating multiple signaling pathways [28]. AMPK-Drp1 axis is involved in Sirt3-mediated attenuation of cardiac injury after infarction [29]. Activation of AMPK by Ligustilide induces Drp1-mediated mitochondrial fission and mitophagy leading to protection of nerve cell apoptosis, whereas knockdown of AMPK*α*2 attenuates LIG-mediated beneficial effect [30]. Moreover, pharmacological activation of AMPK also ameliorates endothelial dysfunction and ER stress by suppression of Drp1 activity [31]. ROS is mainly produced as a by-product of mitochondrial metabolism and is a critical contributor to I/R-induced mitochondrial dysfunction and cardiac injury [32]. Previous studies showed that activation of AMPK inhibits mitochondrial ROS production via multiple signaling pathways, such as NOX4, NF-*κ*B/NLRP3, SIRT1-PGC-1*α*, and OPA1 during I/RI [33–35]. Here, our results indicated that RGDS-mediated activation of LKB1-AMPK signaling remarkably reduced ROS, 8-OHdG, and Drp1 levels but increased Mfn1/2 levels (Figures 4(b), 4(c), and 6(a)), suggesting that inhibition of Fn1 can activate LKB1-AMPK signaling to attenuate mitochondrial dysfunction and oxidative stress in I/R hearts.

Following myocardial I/RI, cardiac fibroblasts play important roles in inflammatory and fibrotic process. I/R could increase ROS production and potassium efflux in cardiac myofibroblasts, which in turn activate inflammasomes and subsequent IL-1*β* release, leading to initiation of inflammatory response and recruitment of macrophages and neutrophils in the ischemic heart. Furthermore, inflammatory cytokines can stimulate myofibroblast activation and cause excessive collagen accumulation resulting in cardiac fibrosis [36, 37]. Interestingly, several studies show that short-time I/R (2-24 h) can significantly increase expression of collagen I/III (1.5-fold) and fibrotic area (about 15-25-fold) in the myocardial tissues of rats or mice compared with sham control [38–40], suggesting that increased collagen production is an early event during myocardial I/RI. Consistent with these data, our results further confirmed that I/R for 24 and 72 h also markedly increased expression of cardiac collagen I, collagen III, and ɑ-SMA and fibrotic area compared with sham control, and this effects were greatly inhibited in RGDS-treated hearts (Figures 4(d) and 4(e)). Notably, AMPK plays an important role in myocardial fibrosis and inflammation. For example, activation of AMPK inhibits cardiac fibrosis through hepatocyte nuclear factor 4 alpha (HNF-4*α*)-TGF-*β*1 signaling [41]. Pharmacological activation of AMPK reduces the inflammatory response via blocking NF-*κ*B during hypoxia and reoxygenation condition [42]. Consistent with these findings, our results indicated that RGDS treatment markedly activated LKB1-AMPK signaling, which inhibited I/R-induced activation of TGF-*β*1 and NF-*κ*B (p-P65) pathways, thereby leading to suppression of inflammation and fibrosis in I/R hearts (Figures 4(f) and 6(a)), showing that blocking Fn1 improves myocardial I/RI partially via LKB1-AMPK-mediated inhibition of inflammation and fibrosis.

## 5. Conclusion

This study provides new evidence supporting the hypothesis that inhibition of Fn1 attenuates myocardial I/RI and myocyte apoptosis, possibly by activating the AMP-LKB1-AMPK-mediated signaling pathways. However, further experiments are warranted to understand the mechanisms underlying Fn1 inhibition of LKB1-AMPK signaling and test whether Fn1 targeting represents a novel target for intervention of ischemic heart diseases in other animals.

## Figures and Tables

**Figure 1:** Ischemia/reperfusion injury upregulates Fn1 expression in mouse heart tissues and STEMI patients. (a) qPCR analysis the mRNA expression of Fn1 (*n* = 4 per group). (b) Immunoblotting analysis of Fn1 protein levels in the I/R heart (upper). Quantification of the protein band (bottom, *n* = 4). GAPDH as an internal control. (c) Fn level in blood samples of normal controls (*n* = 30) and STEMI patients (*n* = 30). Data are expressed as mean ± SEM. ^∗^*P* < 0.05; ^∗∗^*P* < 0.005; ^∗∗∗^*P* < 0.001; ^∗∗∗∗^*P* < 0.0001 versus the sham or normal control.

**Figure 2:** Administration of Fn1 inhibitor alleviated I/R-induced cardiac dysfunction. (a) Fn1 inhibitor RGDS structure. (b) Schematic representation of the experimental protocol. Male wild-type mice (*n* = 8 per group) were treated with Fn1 inhibitor RGDS and then subjected to myocardial I/R for 24 or 72 hours. (c) Echocardiographic images of the left ventricle (top). (d) Quantification of EF%, FS%, LVIDs, and LVIDd (bottom, *n* = 8 per group). Data are expressed as mean ± SEM. ^∗∗∗^*P* < 0.001; ^∗∗∗∗^*P* < 0.0001 versus the sham-operated group; ^##^*P* < 0.01; ^###^*P* < 0.001, ^####^*P* < 0.0001 versus I/R 24 h; ^&&^*P* < 0.01; ^&&&^*P* < 0.001, ^&&&&^*P* < 0.0001 versus I/R 72 h.

**Figure 3:** Administration of Fn1 inhibitor attenuated I/R-induced cardiac infarction and apoptosis. (a) Representative images of TTC and Evens blue staining of myocardial sections after I/RI (top). TUNEL (red), *α*-actinin (green), and DAPI (blue) staining of the myocardial sections (middle). (b) Ratios of area at risk (AAR)/left ventricular (LV) area and infarct size/area at risk (AAR), and quantification of the TUNEL-positive nuclei (bottom, *n* = 5 per group). Scale bar: 5 mm or 20 *μ*m. (c) Immunoblotting analysis of the protein levels of Bcl2, Bax, and cleaved caspase-3 proteins (left) and quantification of the relative protein levels (right, *n* = 4 per group). Data are expressed as mean ± SEM. ^∗∗∗^*P* < 0.001; ^∗∗∗∗^*P* < 0.0001 versus the sham-operated group; ^##^*P* < 0.01; ^###^*P* < 0.001, ^####^*P* < 0.0001 versus saline I/R 24 h; ^&&^*P* < 0.01; ^&&&^*P* < 0.001, ^&&&&^*P* < 0.0001 versus saline I/R 72 h.

**Figure 4:** Administration of Fn1 inhibitor attenuated I/R-induced cardiac inflammation, oxidative stress, and fibrosis. (a) Immunohistochemical staining of myocardial sections with anti-Mac-2 antibody (left), and quantification of Mac-2-positive macrophages (right, *n* = 5). (b) DHE (bottom) staining of myocardial sections (left), and quantification of the ROS level (right, *n* = 5). (c) Masson trichrome's staining of myocardial sections (left), and quantification of the relative fibrotic area (right, *n* = 5). (d) Measurement of 8-OHdG level in the heart (*n* = 5). (e) qPCR analysis of the mRNA levels of collagen I and collagen III in the heart (*n* = 6). (f) Immunoblotting analysis of the protein levels of TGF-*β*1, p-P65, and P65 (left) and quantification of the relative protein levels (right, *n* = 4 per group). GAPDH as an internal control. Data are expressed as mean ± SEM. ^∗∗∗^*P* < 0.001; ^∗∗∗∗^*P* < 0.0001 versus the sham-operated group; ^##^*P* < 0.01; ^###^*P* < 0.001, ^####^*P* < 0.0001 versus saline I/R 24 h; ^&&^*P* < 0.01; ^&&&^*P* < 0.001, ^&&&&^*P* < 0.0001 versus saline I/R 72 h.

**Figure 5:** Administration of Fn1 inhibitor restored the I/R-induced decrease in glucose and fatty acid uptake in I/R hearts. (a) Representative PET images of axial (top), coronal (middle), and sagittal (bottom) cardiac sections with [^18^F]-FDG in mice at 24 or 72 hours after I/RI (left) and quantification of the left ventricular (LV)/blood standard uptake values (SUV) for saline or RGDS-treated mice (right, *n* = 3), showing myocardial glucose uptake. (b) Representative PET images: axial (top), coronal (middle), and sagittal (bottom) cardiac sections with [^18^F]-FTHA in mice at 24 or 72 hours after I/RI (left) and quantification of the LV/blood SUV for saline or RGDS-treated mice (right, *n* = 3), showing myocardial fatty acid (FA) uptake. Data are expressed as mean ± SEM. ^∗∗∗^*P* < 0.001; ^∗∗∗∗^*P* < 0.0001 versus the sham-operated group; ^##^*P* < 0.01; ^###^*P* < 0.001, ^####^*P* < 0.0001 versus saline I/R 24 h; ^&&^*P* < 0.01; ^&&&^*P* < 0.001, ^&&&&^*P* < 0.0001 versus saline I/R 72 h.

**Figure 6:** Administration of Fn1 inhibitor increased the AMP/ATP ratio and activated LKB1-AMPK signaling in I/R hearts. (a) Immunoblotting analysis of the protein levels of p-LKB1 (S428), LKB1, p-AMKP (T172), AS160, GLUT4, Mfn1, Mfn2, (left), p-Drp1 (S616), and Drp1. GAPDH as an internal control. (b) The quantification of the relative protein levels (right, *n* = 4 per group). (c) Measurement of AMP and ATP contents and the ratio of AMP/ATP (*n* = 5). Data are expressed as mean ± SEM. ^∗∗∗^*P* < 0.001; ^∗∗∗∗^*P* < 0.0001 versus the sham-operated group; ^##^*P* < 0.01; ^###^*P* < 0.001, ^####^*P* < 0.0001 versus saline I/R 24 h; ^&&^*P* < 0.01; ^&&&^*P* < 0.001, ^&&&&^*P* < 0.0001 versus saline I/R 72 h.

**Figure 7:** A working model of fibronectin 1 mediating myocardial I/RI. In response to I/R stress, Fn1 expression is upregulated and inhibits activation of LKB1-AMPK signaling, which reduces glucose and fatty acid uptake and promotes cardiac mitochondrial fission, apoptosis, fibrosis, and inflammation via regulating Drp1-Mfn1/2 balance, TGF-*β*1 and NF-*κ*B signaling pathways, thereby leading to cardiac injury. Conversely, blocking Fn1 reverses these effects.

**Table 1:** List of primary antibodies used in immunoblotting analysis.

Antibody	Species	Dilution	Company
Fn1	Human, mouse, rat	1 : 2000	Proteintech (15613-1-AP)
Bcl2	Human, mouse, rat	1 : 2000	Proteintech (26593-1-AP)
Bax	Human, mouse, rat	1 : 2000	Proteintech (50599-2-Ig)
Cleaved caspase-3	Human, mouse, rat	1 : 2000	Proteintech (19677-1-AP)
Mfn-1	Human, mouse, rat	1 : 2000	Proteintech (13798-1-AP)
Mfn-2	Human, mouse, rat	1 : 2000	Proteintech (12186-1-AP)
GLUT4	Human, mouse, rat	1 : 1000	Proteintech (66846-1-Ig)
Phospho(p)-LKB1(S428)	Human, mouse, rat	1 : 1000	Arigobio (ARG42362)
LKB1	Human, mouse	1 : 1000	Arigobio (ARG59080)
AS160	Human, mouse, rat	1 : 2000	Abcam (ab189890)
p-AMPK (T172)	Human, mouse, rat	1 : 1000	Cell Signaling Technology (#2535)
AMPK	Human, mouse, rat	1 : 3000	Cell Signaling Technology (#2532)
p-Drp1(S616)	Human, mouse, rat	1 : 1000	Cell Signaling Technology (#3455S)
Drp1	Human, mouse, rat	1 : 3000	Cell Signaling Technology (#5391S)
TGF-*β*1	Human, mouse, rat	1 : 1000	Cell Signaling Technology (#3711S)
p-P65	Human, mouse, rat	1 : 1000	Cell Signaling Technology (#3039)
P65	Human, mouse, rat	1 : 3000	Cell Signaling Technology (#4764)
GAPDH	Human, mouse, rat	1 : 5000	Cell Signaling Technology (#5174)

**Table 2:** Baseline characteristics of normotensive control subjects and STEMI patients.

Parameters	Normotensive controls (*n* = 30)	STEMI patients (*n* = 30)	*P* value
Age, y	49.433 ± 1.315	62.677 ± 1.975^∗∗∗^	<0.001
Male, *n* (%)	11 (36.667)	24 (77.419)	0.009
LVEF, %	60.967 ± 0.320	49.419 ± 1.251^∗∗∗^	<0.001
Creatine kinase-MB, U/l	0.980 ± 0.130	114.956 ± 29.513^∗∗∗^	<0.001
Cardiac troponin I, *μ*g/ml	0.013 ± 0.004	148.272 ± 27.263^∗∗∗^	<0.001
Systolic blood pressure, mmHg	123.733 ± 2.372	120.226 ± 3.813	0.368
Heart rate, bpm	66.967 ± 0.913	73.903 ± 2.756^∗^	<0.013
Total cholesterol, mmol/l	0.995 ± 0.076	4.753 ± 0.174^∗∗∗^	<0.001
LDL cholesterol, mmol/l	2.809 ± 0.118	2.713 ± 0.116	0.668
HDL cholesterol, mmol/l	1.470 ± 0.060	1.005 ± 0.040^∗∗∗^	<0.001
Triglycerides, mmol/l	5.247 ± 0.161	1.496 ± 0.116^∗∗∗^	<0.001
Creatinemia, umol/l	60.333 ± 2.060	72.452 ± 3.251^∗∗^	0.003
Uric acid, umol/l	280.633 ± 11.697	372.226 ± 19.274	<0.001
Fasting blood glucose, mmol/l	5.052 ± 0.126	5.968 ± 0.510^∗∗∗^	0.093
Platelet, (10^9^/l)	245.533 ± 8.702	238.742 ± 12.152	0.729
White blood cell count, (10^9^/l)	5.567 ± 0.281	10.964 ± 0.555^∗∗∗^	<0.001
Fibronectin 1, (ng/ml)	1.338 ± 0.029	2.614 ± 0.346^∗∗^	<0.001

**Table 3:** Results of the multivariable logistic regression models of Fn1 on STEMI.

Model	Odds ratios (95% CI)	*P* value
Plasma Fn1 protein levels (pg/ml)	23.683 (2.007-45.359)	0.032

All models adjusted for age, systolic blood pressure, HDL cholesterol, creatinemia, fasting blood glucose, platelet, and uric acid. CI: confidence interval; HDL: high-density lipoprotein.

## Data Availability

The data used to support the findings of this study are included in the article.
